# A homozygous missense mutation of *WFS1* gene causes Wolfram's syndrome without hearing loss in an Iranian family (a report of clinical heterogeneity)

**DOI:** 10.1002/jcla.23358

**Published:** 2020-05-17

**Authors:** Shahram Torkamandi, Somaye Rezaei, Reza Mirfakhraie, Sahar Bayat, Samira Piltan, Milad Gholami

**Affiliations:** ^1^ Department of Medical Genetics and Immunology Faculty of Medicine Urmia University of Medical Sciences Urmia Iran; ^2^ Department of Neurology Imam Khomeini Hospital Urmia University of Medical Sciences Urmia Iran; ^3^ Department of Medical Genetics Faculty of Medicine Shahid Beheshti University of Medical Sciences Tehran Iran; ^4^ Department of Medical Genetics Faculty of Medicine Tabriz University of Medical Sciences Tabriz Iran; ^5^ Molecular and Medicine Research Center Arak University of Medical Sciences Arak Iran; ^6^ Department of Biochemistry and Genetics School of Medicine Arak University of Medical Sciences Arak Iran

**Keywords:** gene, homozygous, mutation, *WFS1*, Wolfram's syndrome

## Abstract

**Background:**

Wolfram's syndrome (WFS) is a hereditary (autosomal recessive) neurodegenerative disorder. The clinical features are related to diabetes insipidus, diabetes mellitus, optic atrophy, and deafness (DIDMOAD) with other variable clinical manifestations. Pathogenic variants in the *WFS1* gene, encoding wolframin, are known to be the main cause of Wolfram's syndrome. In this study, we present the clinical and genetic characteristics of two WFS patients from an Iranian family.

**Methods:**

The mutation screening was performed by polymerase chain reaction (PCR) followed by direct Sanger sequencing of all exons from two affected WFS.

**Results:**

The complete Sanger sequencing of the *WFS1* gene detected a homozygous missense variant, c.2207G>A (p.Gly736Asp), in the eighth exon of the *WFS1* gene. Both cases developed all the major symptoms of the disease, interestingly, except hearing loss.

**Conclusions:**

Because of the rarity and clinical heterogeneity of WFS, the molecular genetic assay is essential to confirm the diagnosis and management of the WFS patients.

## 1 INTRODUCTION

Wolfram's syndrome (WFS; OMIM#222300) is a rare, hereditary, and neurodegenerative disease with an autosomal recessive pattern of inheritance.^1^ The estimated prevalence of Wolfram's syndrome is 1 in 68,000 to 770,000 in overall population worldwide.^2^, ^3^, ^4^ WFS is described by the juvenile onset of diabetes mellitus and optic atrophy (at age < 16 years), and associated with sensorineural hearing loss, progressive neurologic abnormalities (peripheral neuropathy, cerebellar ataxia, psychiatric illness, dementia, and urinary tract atony) and other endocrine abnormalities.^5^ According to the literature, genetic variants in the *WFS1* are responsible for disease development.^6^, ^7^ The gene, located at 4p16.1, contains eight exons and encodes a transmembrane 890‐amino acid protein, called wolframin.^8^ The wolframin protein is expressed in several tissues (pancreas, lung, liver, heart, bone, muscle, brain, and kidney).^9^ Its function in the endoplasmic reticulum (ER) that is involved in protein production, processing, and transport, maintaining homeostasis of the amount of intracellular calcium.^8^ Perturbations in ER function result in the accumulation of misfolded proteins, a state entitled ER stress,^10^ and result in WFS. Several mutations have been reported in *WFS1* gene, mostly located in the exon 8, including missense, insertion, deletion, and splice site mutations in the form homozygote and compound heterozygote.^11^ The purpose of the present study was mutational analysis of the *WFS1* gene and investigation of the genotype‐phenotype correlation in a consanguineous Iranian family with Wolfram's syndrome.

## 2 MATERIALS AND METHODS

The current study was approved by the Ethics Committee of the Arak University of Medical Sciences (IR.ARAKMU.REC.1398.115). After obtaining written informed consent, two affected and four unaffected subjects from the family members of consanguineous Iranian with WFS were enrolled in this present study. The research related to human use has been complied with all the relevant national regulations, institutional policies, and in accordance the tenets of the Helsinki Declaration, and has been approved by the authors' institutional review board or equivalent committee. The pedigree of the WFS family with an autosomal recessive pattern of inheritance is shown in Figure 1A.

**FIGURE 1:** A, The family pedigree of Wolfram's syndrome. B and C, The mutation status of *WFS1* (c.2207G>A) was identified by the Sanger sequencing (marked with a red box), the patients (IV‐1 and IV‐5) were homozygous for c.2207G>A and her parents (III‐1 and III‐2), and brothers (IV‐4) were in the heterozygous state. D, Multiple sequence alignment demonstrates high conservation of the p.G736 residue (marked with a black box)

Genomic DNA was extracted from peripheral blood samples obtained from all subjects using the salting‐out method. Forward and reverse primers (Table 1) were designed by the Primer‐BLAST (https://www.ncbi.nlm.nih.gov/tools/primer‐blast/). Amplification of non‐coding, coding (exons 1‐8), and flanking intronic regions of the *WFS1* gene was performed with PCR on a thermal cycler (Peqlab). The PCR reaction contained 17 μL Taq DNA Polymerase Master Mix Red (Ampliqon, Denmark), 0.5 μL of each of the primers (10 PM), 21 μL ddH_2_O, and 1.5 μL DNA. Thermal cycling conditions include a primary denaturation step at 95°C for 6ʹ; 33 cycles of three steps: denaturation at 95°C for 32″, annealing (temperature and time variable according to Table 1), and extension at 72°C for 25″, and a final extension step at 72°C for 4ʹ. The PCR products were subjected to direct Sanger sequencing using an ABI PRISM 3130XL (Applied Biosystems). Finally, the sequencing results were aligned with a reference sequence in NCBI (https://blast.ncbi.nlm.nih.gov) using the Chromas software (version 2.6.2). The segregation analysis of the *WFS1* mutation was performed in the family.

**TABLE 1:** Primers sequences used for PCR‐Sanger sequencing

Gene	Exon	Sequence	PCR products	Annealing temperature/time
*WFS1*	1	F: 5′‐CGCTCGGAAACTTTCGCTGT‐3ʹ R: 5ʹ‐TCCAACTTCGGGGACCTTG‐3ʹ	553 bp	61°C/20ʺ
	2	F: 5ʹ‐TGTATGGAGTGTCTGGCAGC‐3′ R: 5′‐ATGCTGAACTGCAGAGGACC‐3′	470 bp	61°C/20ʺ
	3	F: 5′‐GCAAACAGTGGCTTTCTGGG‐3′ R: 5′‐GAACATGGGCACCCTACCAA‐3′	434 bp	60°C/20ʺ
	4	F: 5′‐ACCGTGTTTTGAGGAGCGAG‐3′ R: 5′‐CAACAGCATCACCAGCGTTAG‐3′	453 bp	60°C/20ʺ
	5	F: 5′‐TGTCCATGCATCCTTCCCTG‐3′ R: 5′‐CAAAATGCCACCCACACACC‐3′	541 bp	61°C/20ʺ
	6	F: 5′‐CAGAACGTAGGATGCCCCTG‐3′ R: 5′‐CTACTCCCAGCGTCCAGAAC‐3′	423 bp	60°C/20ʺ
	7	F: 5′‐CAGGGAAGGGTTTCCTCCAC‐3′ R: 5′‐ATGACCCAAAGGTACCAGCG‐3′	442 bp	60°C/20ʺ
	8‐1	F: 5′‐TTCCTTTTGCCCAGAGGCAG‐3′ R: 5′‐ACACCACATGAAGCACACCA‐3′	861 bp	61°C/25ʺ
	8‐2	F: 5′‐GCTACCTTGTGCCCTACCTG‐3′ R: 5′‐AGCACGATGTCCTTGGTGAC‐3′	826 bp	61°C/25ʺ
	8‐3	F: 5′‐ACATCAAGAAGTTCGACCGC‐3′ R: 5′‐ACACCGGAACCTCCTAGTCT‐3′	670 bp	59°C/20ʺ

We searched in the population databases (dbSNP, ExAC, 1000 Genomes, and gnomAD) and disease databases (ClinVar and HGMD) to exclude the normal variations and investigate the novelty of the mutation. Predicted pathogenicity of the candidate variant was investigated in silico by predictive algorithms, including HOPE (https://www3.cmbi.umcn.nl/hope/), SIFT (https://sift.bii.astar.edu.sg/), Poly‐Phen2 (http://genetics.bwh.harvard.edu/pph2/), MutationTaster (http://www.mutationtaster.org/), and CADD (http://cadd.gs.washington.edu).

We performed a full three‐dimensional (3D) structural modeling of the WFS1 protein with the based on 5IJO protein configuration in the Protein Data Bank (PDB) using I‐TASSER online software (Figure 2B). Then computational visualization of the protein residues was done by PyMOL script (https://pymol.org/2/). Finally, we used MetaDome software to determine the tolerance of the mutated residue for better interpret of the variant with unknown significance. MetaDome mapped population variations from the gnomAD and pathogenic variants from ClinVar, and allowed to create genetic intolerance regions at the amino acid resolution for human protein domains.

**FIGURE 2:** A, The hypothetical schematic transmembrane structure of wolframin. The red circle located in ER lumen depicted pathogenic mutation residue. B, Overall full cartoon wolframin model was created by I‐TASSER modeling using PDB (5IJO). C and D, The magnified view of the normal and mutated residues at location 736 of wolframin protein are revealed as sticks (glycine as normal and aspartate as mutant residue). The yellow dash indicated hydrogen bond, and aspartate736 forms different hydrogen bond compared to glycine 736. E, A tolerance landscape for wolframin was produced by MetaDome web server, the mutations situated in the intolerant regions based on a missense‐over‐synonymous ratio

## 3 RESULTS

### 3.1 Clinical description

The probands, two male (IV‐1 and IV‐5), were born to healthy Iranian consanguineous parents originating from a Bakhtiari ethnicity (Figure 1A). They have two healthy brothers (IV‐3 and IV‐4) and an unaffected sister (IV2) who died because of the single ventricle in the sixth month of life. Wolfram's syndrome was not present in the family ancestry.

Patient IV‐1 is a 40‐year‐old man with diabetes (insipidus and mellitus) identified before the age of 22 years, monitored by reduced visual acuity at 24 years old with a history of mitral valve prolapse, neurogenic bladder, polyuria, and urinary incontinence. Ophthalmological investigation revealed a reduction of visual acuity and loss of color vision owing to bilateral optic atrophy.

Patient IV‐5, a 28‐year‐old man, has a history of diabetes (insipidus and mellitus) detected before the age of 8 years and monitored by the reduced visual acuity at 12 years old with a history of dextrocardia, pulmonary artery stenosis, neurogenic bladder, polyuria, and urinary incontinence; after that both patients showed signs of diabetes and reduced visual acuity, and the clinical geneticist refers them to an otolaryngologist for exact audiological examinations including pure‐tone audiometry (0.25‐8 kHz) and tympanometry. Interestingly, the results of all these audiological tests were normal in both patients. Besides, during these years, the patients have been evaluated several times for audiometry and have had no problems so far.

### 3.2 Mutational analysis

One homozygous missense variant, Figure 1C, was found in the exon 8 of both affected siblings as c.2207G>A. The parents (III‐1 and III‐2) and healthy brothers (IV‐4) were heterozygous, for the mutation (Figure 1B), and did not present any symptoms of WFS. Besides, the other brother (IV‐3) was homozygous for the wild‐type allele. The c.2207G>A alteration leads to the exchange of glycine (the most flexible of all residues) to aspartic amino acid at the position 736 in the protein product of wolframin (p.G736D) (Figure 2A). This variant has been previously described in the homozygous form in a single individual from a consanguineous marriage and was considered as a variant with uncertain significance, the clinical characteristics of this patient include diabetes mellitus, optic atrophy, and diabetes insipidus, and the hearing status was not determined (https://www.ncbi.nlm.nih.gov/clinvar/variation/618493/).

According to the HOPE program, the wild‐type and mutant residue charge were neutral versus negative, respectively. Furthermore, the wild‐type residue is more hydrophobic than the mutant residue, and this mutation decreases the stability of the protein structure with Confidence Score: −0.602 (probably damaging). The new amino acid affects the α‐helix structure by creating different hydrogen bonds (Figure 2C,D). The p.G736D was predicted to be highly deleterious using the SIFT and PolyPhen programs. Also, MutationTaster predicted this mutation to be “disease‐causing” variant, and with 29.5 CADD Phred score, which is over the deleterious threshold. Multiple sequence alignment exhibited that p.Gly736 residue in WFS1 is evolutionarily conserved across different species (Figure 1D), representing its importance in the function of WFS1 protein. MetaDome software also showed that this residue is an intolerance region for any mutation (Figure 2E). Furthermore, according to the HOPE, the mutation is located within a section of residues that is repeated in the protein named as lumenal. Under this conservation information, this alteration is most likely damaging to the wolframin protein.

## 4 DISCUSSION

Up to the present time, more than 219 distinct mutations in the *WFS1* gene have been reported worldwide in the HGMD database (http://www.hgmd.cf.ac.uk/ac/gene.php?gene=WFS1). Genetic studies in WFS subjects have recognized a wide variety of mutations, including frameshift, stop codon and splice site, and missense mutations.^12^ These mutations are responsible for inactivating of WFS1 protein due to their loss‐of‐function effect.^12^ Different types of mutations positioned in the hydrophilic C‐terminal part of the WFS1 protein underlines the efficient importance of the C‐terminus.

In our survey, we found a probably pathogenic missense mutation (c.2207G>A) in an Iranian family with significant consequences on *WFS1* configuration and function. Previous studies have reported that the residue G736 is a hot spot mutation point (G736R, G736D, G736S).^13^ Our description of the c.2207G>A (p.G736D) mutation in *WFS1* is the second description of a mutation related with WFS in an Iranian family and is the third report worldwide.^14^, ^15^ However, two previous studies did not investigate parental segregation of the mutation and carrier situation.^14^, ^15^ Furthermore, in our study, the patients revealed no signs of hearing loss, while in the previous survey, loss of auditory acuity in both ears was reported at the age of 16.^14^ Moreover, the hearing status was not determined in a Japanese patient.^15^ The clinical heterogeneity between the patients with the same mutation may be partly due to the effects of modifier genes and the natural variants in the *WFS1* gene. Consistently, the effects of modifier genes and alleles on the clinical heterogeneity have been reported in previous studies.^16^, ^17^ Interestingly, similar to our research, it was recently reported that c.376G>A mutation in the exon 4 did not result in the hearing loss in an Iranian patient with WFS.^18^

In one study, subjects with WFS were subdivided into three groups consistent with the predicted functional consequences of each mutation.^15^ Group 1 had frameshift and/or deletion/insertion mutations in homozygote pattern with predicted whole loss of function and early onset of optic atrophy and diabetes mellitus. Group 2 included subjects carrying single amino acid insertions and/or missense mutations in a homozygote pattern with partial loss of function with mild ages of onset of optic atrophy and diabetes mellitus. The group 3 were individuals with compound heterozygous mutations and an average ages of onset of diabetes mellitus and optic atrophy. According to the mentioned classification, the c.2207G>A mutation falls into the group 2, and the age of onset of diabetes mellitus and optic atrophy in our subjects was similar to this category. So, these differences in the age of onset may be correlated with special effects of such alterations on WFS1 protein function.

Management of Wolfram's syndrome is symptomatic and supportive. It involves a multidisciplinary work to manage the different features of this disorder such as insulin therapy (for diabetes mellitus), vasopressin (for diabetes insipidus), and hearing aids or cochlear implants (for hearing loss).^5^ Early diagnosis through genetic testing can help to dismiss the symptoms, avoiding future complications and improving the quality of life for WFS subjects.

In conclusion, we found a missense mutation which was shared between the considered patients. Altogether, according to previous studies, there was not sufficient evidence to classify c.2207G>A as a particular pathogenic variant. The evidence from the present study, such as population data frequency, computational and bioinformatics analysis, and segregation of the mutant variant in the family, classified the c.2207G>A as a pathogenic variant consistent with ACMG standards for the interpretation of sequence variants. To confirm the function of c.2207G>A mutation and its effect on disease development, additional functional studies are necessary. Also, the molecular survey of further Iranian WFS patients is required to conclude the origin and frequency of the mutation. Such researches are useful for carrier detection, genetic counseling, genotype‐phenotype correlation investigation, and prenatal diagnosis.

## CONFLICT OF INTEREST

Authors do not have any conflict of interest to disclose.
